# MFOC-CliqueNet: A CliqueNet-Based Optimal Combination of Multidimensional Features Classification Method for Large-Scale Laser Point Clouds

**DOI:** 10.1155/2022/2446212

**Published:** 2022-08-11

**Authors:** Lei Wang, Zhiyong Zhang, Xiaonan Li, Yueshun He

**Affiliations:** ^1^Jiangxi Key Laboratory of Cybersecurity Intelligent Perception, East China University of Technology, Nanchang 330013, Jiangxi, China; ^2^School of Information Engineering, East China University of Technology, Fuzhou, China

## Abstract

As large-scale laser 3D point clouds data contains massive and complex data, it faces great challenges in the automatic intelligent processing and classification of large-scale 3D point clouds. Aiming at the problem that 3D point clouds in complex scenes are self-occluded or occluded, which could reduce the object classification accuracy, we propose a multidimension feature optimal combination classification method named MFOC-CliqueNet based on CliqueNet for large-scale laser point clouds. The optimal combination matrix of multidimension features is constructed by extracting the three-dimensional features and multidirectional two-dimension features of 3D point cloud. This is the first time that multidimensional optimal combination features are introduced into cyclic convolutional networks CliqueNet. It is important for large-scale 3D point cloud classification. The experimental results show that the MFOC-CliqueNet framework can realize the latest level with fewer parameters. The experiments on the Large-Scale Scene Point Cloud Oakland dataset show that the classification accuracy of our method is 98.9%, which is better than other classification algorithms mentioned in this paper.

## 1. Introduction

The development and advancement of 3D scanning technology have significantly improved the measurement efficiency and accuracy of 3D laser point cloud data. The volume of 3D point cloud data is growing at an unprecedented rate. This also makes the processing, analysis, and understanding of massive 3D point cloud data become a new research hotspot in the field of artificial intelligence. Its application prospects are very broad such as photogrammetry, remote sensing, cultural relics protection, autonomous driving, and robot vision. In the process of automatic analysis and processing of 3D point cloud data for large scenes, the point cloud classifications are the basic steps, which have a great impact on subsequent higher level operations. However, due to the self-shielding or self-shielding characteristics of point clouds between different 3D objects in large-scale scenes, the research and application of 3D point cloud classification are challenging.

In recent years, many researches have done a lot of research on multiobject classification in large-scale 3D point cloud data. The DBSCAN algorithm is used to effectively and accurately segment the outdoor large scene point cloud, and then classified the point cloud based on the segmentation result [1]. However, when using DBSCAN algorithm to cluster ungrounded point clouds, some point clouds are not continuous due to the obstacles of 3D objects, resulting in oversegmentation and other phenomena in clustering. To solve this problem, the author proposes a strategy of large-scale including small-scale and proximity fusion, but this method cannot split two closely connected objects, which will affect the point cloud classification results in special scenes. RangNet++ [2] uses the distance image as the intermediate representation; it projects the 3D point cloud onto the front view and compensates for the information loss caused by projection by performing a fast, GPU-based kNN-search postprocessing method. Li et al. [3] distinguish the shapes of plane, cylinder, space body, and sphere mainly by using four features of volume, normal vector, principal direction, and principal curvature. However, these features are more or less affected by occlusion and noise. Although the methods proposed in some papers compensate for the loss of information [3, 4], the 3D shape features they extract are insufficient to describe a complete 3D object.

This paper proposes a 3D point cloud classification architecture based on MFOC-CliqueNet for large scene. Firstly, three-dimensional nearest neighbor optimization is performed based on neighborhood space, and the three-dimensional features of each point are solved based on the adaptive optimal spherical neighborhood. By analogizing the three-dimensional feature extraction method, point clouds are projected onto three two-dimensional planes: *XOY*, *YOZ*, and *XOZ*, and corresponding two-dimensional features are extracted based on two-dimensional adaptive optimal circle neighborhood. Secondly, the optimal combination feature matrix MFOC is obtained by arranging and weighting the two-dimensional and three-dimensional features. Finally, the feature matrix is imported into the CliqueNet to fully learn the features related to the training data, so as to further improve the classification efficiency of large scene point clouds. The main contributions of this paper are as follows:

1. We propose an optimal combination method of point cloud multidimensional features. The 2D and 3D features of the point cloud are arranged, weighted, and combined, and the optimal combined feature matrix MFOC is constructed.
2. MFOC can better describe the local and contextual global structure of the point cloud in large scale. And it can improve the accuracy of cloud multitarget classification in complex large-scale scenic.
3. In this paper, CliqueNet, a cyclic convolution network, is apply to the classification of 3D point cloud data in large scenes for the first time, and we propose a large-scene 3D point cloud classification architecture based on MFOC-CliqueNet.
4. We conducted experiments on the Oakland data set. And the experimental results show that the method achieves a good classification accuracy in large-scale point cloud.

## 2. Related Works

The deep learning algorithm was first applied in two-dimensional image processing, and achieving outstanding performance and mature technology. For example, AlexNet [4] applied numerous methods to improve model performance, such as the first use of ReLU nonlinear activation function and the first use of dropout and the regularization of the network through massive data enhancement. VGG-Net [5] proposed by Oxford University has a smaller convolution kernel and deeper level than AlexNet, which further improves the parameter efficiency. GoogLeNet [6] contains a very efficient Inception module; it does not use a fully connected network as VGG-Net does, so the amount of parameters is very small. The significant work of ResNet [7] is to solve the problem of gradient disappearance during back propagation, so it can train very deep networks without adding a classification network in the middle like GoogLeNet. Although ResNet is very efficient, not every layer of such a deep network is effective, these redundant convolutional layers and feature maps will reduce the parameter efficiency of the model. To this end, Huang et al. [8] proposed DenseNet, the goal of this network is to improve the efficiency of information flow and gradient flow between network layers and to improve the efficiency of parameters. This structure ensures that each layer can directly access the gradient from the loss function, so it can train very deep networks. Although DenseNet has few parameters, the memory usage is very large. Yang et al. [9] proposed CliqueNet, which has achieved good results in the two-dimensional image recognition task. Its advantage is that it not only has the prequel part but also optimizes the feature maps of the previous level according to the output of the latter level. This architecture is inspired by the cyclic structure and attention mechanism, that is, the feature maps output by the convolution can be reused, and the refined feature maps will pay attention to more important information. Within the same Clique module, there are forward and reverse connections between any two layers, which also enhances the information flow in the deep network. It has the advantages of parameter amount and calculation amount. Therefore, we introduce the CliqueNet to perform feature learning on the 2D and 3D features of the large-scene 3D point cloud and obtain better classification results.

As the advancement of 3D laser scanning technology, the quality and accuracy of the collected 3D point cloud data have been greatly improved. Therefore, a study of the analysis and processing based on the 3D point cloud data is significant. Many researchers have begun to apply deep learning to 3D point cloud data processing. In order to make 3D point cloud data suitable for 2D convolutional neural networks, 3D point cloud data are usually preprocessed and then input into the network. At present, the main methods to solve the problems of unstructured and disordered point clouds are as follows. (1) Multiview: Representing three-dimensional objects with pictures from different angles, that is, converting 3D CNN into 2D CNN technology for classification and other tasks. The most representative study is MVCNN [10]. The author projects 3D objects through different angles to obtain multiview 2D images to represent 3D objects. However, in the face of complex large-scale scene tasks, a fixed number of multiview images cannot describe all the targets in a three-dimensional large scene well. (2) Volumetric: mainly to solve the problem of disorder of point cloud, by regularizing the 3D point cloud. This method does improve the performance of point cloud classification, but due to its large amount of computation and low resolution of voxel mesh, it takes up a lot of memory and loses local information, it is still not suitable for complex large scenes. There are some representative studies, such as 3D ShapeNets [11], the probability distribution of 3D voxel grid binary variables is used to represent the 3D shape. It learns the joint distribution of input and labels by constructing a convolution DBN. VoxNet [12] is proposed by Maturana and Scherer, which uses semisupervised 3DCNN to process the occupied 3D voxel grid. (3) Point clouds are processed directly: this kind of method directly act on the original point cloud, without any transformation of the original point cloud, and retain their rich location information. Charles et al. [13] proposed PointNet, breaking the tradition for the first time, so that the network can directly handle point cloud, and the author uses symmetric functions to avoid the disorder of point cloud. The feature extraction method of PointNet is to extract a global feature for all point cloud data. Obviously, this is different from the current popular CNN method of extracting local features layer by layer. Inspired by CNN, the author proposed PointNet++ [14], which can extract local features at different scales and obtain deep features through a multilayer network structure. PointConv [15] can construct a multilayer deep convolutional network on a 3D point cloud, this structure can achieve the same translation invariance as 2D convolutional networks, and permutation invariance of point order in point cloud. This type of method has received more and more attention. However, the type of point cloud data used in this method is different from the first two methods; the method is oriented to the 3D point cloud model data, rather than the point cloud data for the large scene.

## 3. Methods

We propose a large-scale 3D point cloud classification architecture based on MFOC-CliqueNet. We construct multidimensional feature optimal combination matrix (MFOC) of the large-scale 3D point cloud, and import CliqueNet cyclic network to the field of 3D point cloud classification for large scene for the first time. First, the “Kd-Tree” algorithm is used to search for 100 nearest neighbors for each point in the large-scene 3D point cloud data set and obtaining the optimal neighborhood adaptive radius based on the method of minimum Shannon entropy [16]. Then the 3D eigenvalues and eigenvectors corresponding to the 3D covariance matrix of the point cloud are calculated based on the optimal neighborhood adaptive spherical radius. Meanwhile, the 3D point cloud was projected to the *XOY*, *YOZ*, and *XOZ* planes to extract the 2D features. Based on the optimal neighborhood adaptive circle radius, we calculate the 2-dimensional eigenvalues and eigenvectors corresponding to the point cloud. However, the simple horizontal random combination of the multidimensional features of the point cloud is not good. Therefore, it is necessary to combine 2D and 3D features according to certain principles to obtain a multidimensional feature matrix. Here, we propose some optimal combination principles:

1. Arranging the 2D projection features diversely to obtain the optimal arrangement features.
2. The 2-D and 3-D features are combined with different weights, and the optimal combination features are obtained according to the specific permutation weighted combination experiment.
3. Finally, the optimal combination of the multidimensional features matrix MFOC is integrated into the CliqueNet to construct the MFOC-CliqueNet to achieve 3D point cloud classification. The MFOC-CliqueNet architecture is illustrated in Figure 1.

In order to better describe the local structure of the large-scale 3D point cloud, this paper adopts the two-dimensional projection feature extraction based on the two-dimensional nearest circular neighborhood and the three-dimensional feature extraction based on the three-dimensional nearest spherical neighborhood, respectively. The characteristic values, characteristics, and geometric features of the matrix based on 3D covariance matrix are extracted using the 3D structure tension [17]. The 3D point cloud is projected to the *XOY*, *YOZ*, and *XOZ* planes, and the 2D structure tensor is used to extract the 2D features of the point cloud.

### 3.1. A Multidimensional Feature Extraction of the Large-Scale 3D Point Cloud

#### 3.1.1. 2D Feature Extraction

Due to the complexity of outdoor cloud objects in three-dimensional scenic area, self-shielding and be shielded of three-dimensional point cloud data are prone to occur, which affects the accuracy of point cloud object classification. If the point cloud is only projected on the *XOY* plane [18], it cannot well describe the three-dimensional spatial characteristics of the nonplanar structure point cloud objects. In response to this situation, we project the point cloud onto the three 2-dimensional planes *XOY*, *YOZ*, and *XOZ* to obtain richer point cloud feature information, as shown in Figure 2:

(1) The representation form of any point cloud in the *XOY* plane is
  (1) $$\begin{array}{c} \left[\begin{array}{cc} x & y \end{array}\right]=\left[\begin{array}{ccc} x & y & z \end{array}\right]\times \left[\begin{array}{ccc} 1 & 0 & 0\\ 0 & 1 & 0\\ 0 & 0 & 0 \end{array}\right]. \end{array}$$
(2) The representation form of any point cloud in the *YOZ* plane is
  (2) $$\begin{array}{c} \left[\begin{array}{cc} y & z \end{array}\right]=\left[\begin{array}{ccc} x & y & z \end{array}\right]\times \left[\begin{array}{ccc} 0 & 0 & 0\\ 0 & 1 & 0\\ 0 & 0 & 1 \end{array}\right]. \end{array}$$
(3) The representation form of any point cloud in the *XOZ* plane is
  (3) $$\begin{array}{c} \left[\begin{array}{cc} x & z \end{array}\right]=\left[\begin{array}{ccc} x & y & z \end{array}\right]\times \left[\begin{array}{ccc} 1 & 0 & 0\\ 0 & 0 & 0\\ 0 & 0 & 1 \end{array}\right]. \end{array}$$

We use the neighborhoods sought by KD-Tree and the neighborhood optimization based on minimizing Shannon entropy to obtain the best adaptive circular neighborhood *r*_*k*_. And then the two-dimensional structure tensor of each point is calculated, and the sum of feature values *s*_2_, value ratio *R*_*λ*,2*D*_, and two-dimensional local point density *D*_2_ was extracted. Therefore, in this paper, we extract *r*_*k*_, *S*_2_, *R*_*λ*,2*D*_, and *D*_2_ from each plane of the *XOY*, *XOZ*, and *YOZ*.

The given point *p*_*k*_(*x*_*k*_, *y*_*k*_) is the *K*-th nearest neighbor of point *P*, and *K* is the optimal adaptive circular neighborhood size parameter of point P, then the radius of the circular neighborhood at point *P* is

(4) $$\begin{array}{c} r_{\text{k}}=\sqrt{{\left(x-x_{k}\right)}^{2}+{\left(y-y_{k}\right)}^{2}}. \end{array}$$

The two-dimensional local point density [19] is

(5) $$\begin{array}{c} D_{2}=\frac{k+1}{\pi r_{k}^{2}}. \end{array}$$

The characteristic value ratio [20] is

(6) $$\begin{array}{c} R_{\lambda ,2D}=\frac{\lambda_{2,2D}}{\lambda_{1,2D}}. \end{array}$$

The sum of the characteristic values is

(7) $$\begin{array}{c} S_{2}=\lambda_{1,1D}+\lambda_{2,2D}, \end{array}$$

*r*_*k*_ is the radius of the optimal adaptive circular neighborhood. *λ*_2,2*D*_ and *λ*_1,1*D*_ are the eigenvalues corresponding to the two-dimensional covariance matrix.

We visualized the projection of the three-dimensional point cloud on the three planes *XOY*, *XOZ*, and *YOZ*.

Comparing the visualizations in the three directions of *XOY*, *YOZ*, and *XOZ* in Figure 3, you can find that the red area in the middle and the blue and red areas on the right of the left view (Figure 3(a)) are all obscured in the rear view (Figure 3(b)). At the same time, the red area on the left side of Figure 3(b) is also missing in Figure 3(a). The top view (Figure 3(c)) is the most severely blocked. Therefore, the single view cannot fully display the complex 3D objects in the large scene. If one direction is projected, the relatively complete 2D feature information of the 3D point cloud data cannot be extracted. Therefore, in this paper, three-dimensional point cloud is projected onto the planes of *XOY*, *XOZ*, and *YOZ*, respectively.

#### 3.1.2. 3D Feature Extraction

Based on the nearest neighbor computed by KD-tree, the eigenvalues and eigenvectors corresponding to the three-dimensional covariance matrix are computed point by point, and then the following features are computed by combining the neighborhood optimization based on the Minimization of Shannon Entropy:

(8) $$\begin{array}{c} C_{\lambda }=\frac{\lambda_{3}}{\lambda_{1}+\lambda_{2}+\lambda_{3}}. \end{array}$$

Dimensional features are linear, planar, and cluster-like attributes:

(9) $$\begin{array}{c} L_{\lambda }=\frac{\lambda_{1}-\lambda_{2}}{\lambda_{1}},\\ P_{\lambda }=\frac{\lambda_{2}-\lambda_{3}}{\lambda_{1}},\\ S_{\lambda }=\frac{\lambda_{3}}{\lambda_{1}}. \end{array}$$

Three-dimensional local point density is as follows:

(10) $$\begin{array}{c} D=\frac{k+1}{\left(4/3\right)\pi r_{k-NN}^{3}}. \end{array}$$

The ball radius is

(11) $$\begin{array}{c} r_{k-NN}=\sqrt{{\left(x_{k}-x\right)}^{2}+{\left(y_{k}-y\right)}^{2}+{\left(z_{k}-y\right)}^{2}}. \end{array}$$

Nearest neighbor tetrahedron volume Q is

(12) $$\begin{array}{c} Q=\frac{1}{6}\left\|\left(\overset{⟶}{pp_{1}}\times \overset{⟶}{pp_{2}}\right)•\overset{⟶}{pp_{3}}\right\|\\ =\left|\begin{array}{ccc} x_{1}-x & y_{1}-y & z_{1}-z\\ x_{2}-x & y_{2}-y & z_{2}-z\\ x_{3}-x & y_{3}-y & z_{3}-z \end{array}\right|. \end{array}$$

*(1) Verticality*. Total variance, anisotropy, feature entropy, and trajectory at this point [21] are as follows:

(13) $$\begin{array}{c} \text{verticality}=1-\left|n_{z}\right|,\\ O_{\lambda }=\sqrt[{3}]{e_{1}e_{2}e_{3}},\\ A_{\lambda }=\frac{e_{1}-e_{3}}{e_{1}},\\ E_{\lambda }=-\sum_{i=1}^{3}e_{i}\ln\left(e_{i}\right),\\ T_{\lambda }=\frac{2}{\pi }\arctan\left(\lambda_{1}+\lambda_{2}+\lambda_{3}\right). \end{array}$$

Given a three-dimensional point *P* (*x*, *y*, *z*), *K* is the nearest neighbor parameter of the point *P*, and *r*_*K*−*NN*_ is the distance from the point *P* to the *K*-th point *p*_*k*_(*x*_*k*_, *y*_*k*_, *z*_*k*_) in its neighborhood. The verticality can distinguish the ground point from the nonground point, and *n*_*Z*_ is the third component of the third-dimensional feature vector of the three-dimensional structure tensor of the current point *P*. *O*_*λ*_, *A*_*λ*_, *E*_*λ*_, and *T*_*λ*_ are local three-dimensional shape features. *e*_1_, *e*_2_, and *e*_3_ are all normalized feature values. *T*_*λ*_ describes the invariant characteristics of points. There are also features related to feature vectors: *v*_*i*1_, *v*_*i*2_, and *v*_*i*3_. *v*_*i*1_ is the maximum distribution direction vector, *v*_*i*3_ is the maximum distribution direction vector, and *v*_*i*2_ is the direction vector perpendicular to *v*_*i*1_ and *v*_*i*3_, they are all three-element vectors. Until now, a total of 29 2D and 3D features has been extracted in this method.

### 3.2. A Large-Scale 3D Point Cloud Classification Based on MFOC-CliqueNet

In this paper, CliqueNet is imported into the 3D point cloud classification of large scenes for the first time, and we propose a large-scene 3D point cloud classification framework based on MFOC-CliqueNet. CliqueNet not only combines the cyclic structure and the attention mechanism but also updates the optimal combination matrix (MFOC) of multidimensional features alternately twice. Then, we can obtain the MFOC with higher feature quality and pass it to the next block. At the same time, it uses a multiscale feature strategy to avoid parameters linear growth, as shown in Figure 4. The TBlock module contains two parts: the Transition layer and the Clique Block. Each Clique Block has output of the *Z*_0_ (MFOC) and stage-II (the second alternately update of the MFOC feature map parameters). These two outputs go through concatenation and then connect to a Global Pooling as part of the prediction. *Z*_0_ represents the input of the first Clique Block, and each subsequent Clique Block input is the result obtained after the output stage-II of the previous block passes through the Transition layer. Thus, each layer is both the input and output from the other layers in Clique Block.

Each Clique Block of CliqueNet contains two stages: the first stage is similar to DenseNet [8], which can be regarded as the initialization process of MFOC; secondly, the input of each convolution operation includes not only the output feature map MFOC of all the previous layers also includes the output feature map $\bar{\text{MFOC}}$ of the subsequent level (Output after the update of Clique Block module).

For the *i*-th layer and *k*-th cycle in the second stage, the alternately updated expression is

(14) $$\begin{array}{c} Z_{i}^{\left(k\right)}=g\left(\sum_{l<i}W_{li}*Z_{l}^{\left(k\right)}+\sum_{m>i}W_{mi}*Z_{m}^{\left(k-1\right)}\right), \end{array}$$

where *k* ≥  2, *W*_*li*_*∗Z*_*l*_ means that the convolution kernel performs a convolution operation on the input feature matrix graph *Z*, and *g* is a nonlinear activation function.

In this paper, the obtained feature matrix *Z*0 is input into CliqueNet, and passes through 64 convolutional layers of 5 × 5 with a stride of 2; then it passes through a pooling layer of 3 × 3 with stride of 2. Each Block is connected by Transition layer, and the network is trained with 250 epochs.

The CliqueNet is set as a three-stage network, including convolution layer, pooling layer and block module. And the CliqueNet node parameter setting at each stage is shown in Table 1. In order to adapt the CliqueNet to the multidimensional feature matrix (32 × 32 × 1) of the large-scale 3D point cloud obtained in this paper, we need to modify the parameters of the original CliqueNet:

1. *K* and *T* in the original network are too large, which is easy to cause over fitting. We reduce *K* and *T* to 12 and 16.
2. Because 3D large-scale point cloud does not need to deal with the three RGB color channels in the color image, we set channel equals 1.
3. Considering the size of the MFOC, we reduce the convolution kernel size of the original CliqueNet, for example, from 7 × 7 to 5 × 5.

## 4. Results

### 4.1. Datasets

The framework proposed is tested on the public Oakland 3D point cloud data set [22]in this paper. The data set is the most widely used, acquired by Mobile Laser Scanner, with marked point cloud data, which is saved in text format. Three real value coordinates are written in each line. The data set represents the urban environment and captured by a mobile platform equipped with a side SICK LMS laser scanner. The data set is divided into training set *X*, verification set *V*, and test set *Y*. Each 3D point is assigned one of five semantic categories, namely wire, pole/trunk, facade, ground, and vegetation. The number of samples in each category is shown in Table 2.

### 4.2. Network Training Details

In this paper, the initial learning rate of the network is 0.001, the total number of training rounds is initially set to 300 epochs, and it adopt a gradual decrease in learning rate. When the number of training rounds is equal to 150 epochs, the learning rate becomes 0.1 of the initial learning rates. The number of rounds is equal to 225 epochs, and the learning rate becomes 0.01 of the initial learning rates. We use the momentum optimization method with a decay rate of 0.9 to train the MFOC-CliqueNet framework. The MFOC-CliqueNet framework in this paper takes about 5 hours to train on the GTX 2060 GPU using TensorFlow.

As shown in Figure 5(a), the initial learning rate is 0.03 (orange line) and the initial learning rate is 0.01 (green line), their test accuracy rates fluctuate greatly and are extremely unstable in the first 150 epochs, even training tests after 150 epochs, the accuracy of the initial learning rate of 0.001 (blue line) has been consistently higher than the previous two. For the choice of optimizer, it can be seen from Figure 5(b) that the performance of the SGD optimizer has the worst accuracy, while the Momentum optimizer performs best, and after several training rounds, its accuracy has been stable at more than 90%.

### 4.3. Multidimensional Features Arrangement

Three-dimensional point clouds are projected onto the *XOY*, *YOZ*, and *XOZ* planes in *X*, *Y*, and *Z* directions, respectively. Four two-dimensional features, *r*_*k*_, *D*_2_, *S*_2_, and *R*_(*λ*, 2*D*)_, are obtained for each plane. In the process of point cloud projection, the result of feature extraction will be affected by occlusion or self-occlusion between objects. Therefore, in this paper, the two-dimensional features extracted from the projected surface are tested in different directions to test the optimal multidimensional feature arrangement.

Initially, the weighted combination ratio of multidimensional features defaults to 3D : 2D = 1 : 1, which means the arrangement of two-dimensional features is added to the original three-dimensional features. Suppose *XOY* = *B*, *YOZ* = *C*, *XOZ* = *D*, there are six different arrangements [*BCD*, *BDC*, *CBD*, *CDB*, *DBC*, *DCB*]. The six arrangements were tested experimentally.

Comparing its experimental results (as shown in Table 3), the overall classification accuracy (OA) of the first three categories is not significantly different, which are all above 97%. However, compared the classification accuracy of each category, the classification efficiency of the DCB sorting is higher than that of other sorting. (Although the classification accuracy of the two types of “poles and vegetation” arranged by DCB was lower than that of other sequences, there was little difference in the comparison accuracy between them.) The comparison accuracy of the other two categories, “wire and facade,” ranked first in DCB, with a large difference. Therefore, we take the

*X*=[(*r*_*k*_, *D*_2_, *R*_(*λ*, 2*D*)_, *S*_2_)_*xoz*_, (*r*_*k*_, *D*_2_, *R*_(*λ*, 2*D*)_, *S*_2_)_*yoz*_, (*r*_*k*_, *D*_2_, *R*_(*λ*, 2*D*)_, *S*_2_)_*xoy*_] as the best arrangement of multidimensional features.

### 4.4. Weighted Combination of Multidimensional Features

On the basis of the previous section, we have obtained the best arrangement and combination of two-dimensional and three-dimensional features. The best arrangement based on two-dimensional characteristics is

(15) $$\begin{array}{c} X=\left[{\left(r_{k},D_{2},R_{\left(\lambda ,2D\right)},S_{2}\right)}_{xoz},{\left(r_{k},D_{2},R_{\left(\lambda ,2D\right)},S_{2}\right)}_{yoz},{\left(r_{k},D_{2},R_{\left(\lambda ,2D\right)},S_{2}\right)}_{xoy}\right]. \end{array}$$

Here, *XOY*, *YOZ*, and *XOZ* represent three two-dimensional projection surfaces, and the three-dimensional features of the point clouds are arranged as follows:

(16) $$\begin{array}{c} Y=\left[L_{\lambda },N_{x},N_{y},N_{z},P_{\lambda },S_{\lambda },M_{x},M_{y},M_{z},O_{\lambda },A_{\lambda },E_{\lambda },T_{\lambda },C_{\lambda },D,Q,V\right]. \end{array}$$

The multidimensional feature weighted combination feature matrix is

(17) $$\begin{array}{c} Z=W_{1}\left[Y\right]+W_{2}\left[X\right], \end{array}$$

where *W*_*i*_ is the weight.

Since the two-dimensional and three-dimensional features have different effects on target classification, the best classification accuracy will not be obtained by simply combining the two-dimensional and three-dimensional features in a 1 : 1 scale. This paper combines the two-dimensional and three-dimensional characteristics of point clouds with the optimal arrangement of different weights to study the validity of point cloud classification accuracy [23]. The experiment shows in Table 4, the 2D features extracted on the 2D projection, and the optimal arrangement DCB obtained from the above section is used for weighted combination of multidimensional features. It can be seen from Table 4 that the overall classification accuracy of each weighted combination has little difference, with the maximum value of 98.22% and the minimum value of 96.90%. Comparing the classification accuracy of the second, fourth, and fifth categories of the first three different weight combinations, it can be concluded that the lower the three-dimensional feature ratio, the lower the classification accuracy.

For the first and third categories, when the combined weight of multidimensional features is 3D : 2D = 0.9 : 0.1, the classification accuracy is the lowest, but the overall classification accuracy is higher than other weight combinations. The experimental results show that the three-dimensional feature is more important than the two-dimensional feature for point cloud classification in large scenes. This paper chooses the weight 3D : 2D = 0.9 : 0.1 to combine multidimensional features to further improve the classification accuracy.

### 4.5. Scaling of Multidimensional Features

The feature combination matrix *Z* can be divided into three parts according to the value of the weight *w*. First, if *w*=1 then it means that the multidimensional features size remains unchanged. Second, if the weight *w* < 1 or *w* > 1 then the features of different dimensions are scaled; and the performance of effective features may be increased by scaling different features. It may also increase the size range between features which is disadvantaged to the fast convergence of gradient descent and thus affects the final classification accuracy. Combining with the multidimensional features matrix designed in our paper, the experiment shows that scaling features of different dimensions with different weight values will affect the classification accuracy of point cloud as shown in Table 5.

Comparing Tables 4 and 5, we reduce and normalize the multidimensional features. The experimental results show that this classification result is better than other amplification weight values. For example, the ratio of 3D : 2D = 0.9 : 0.1 can obtain the best classification accuracy. Through properly scaling and normalization of multidimensional features, the data feature range can be standardized, so that the gradient descent process converges faster.

In summary, the two-dimensional features matrix is the optimal arrangement of *X*={*X*_*D*_, *X*_*C*_, *X*_*B*_} for multidimensional feature weighted combination, and the optimal feature combination matrix *Z* (MFOC) is obtained as the input of CliqueNet:

(18) $$\begin{array}{c} Z=\left[\begin{array}{c} \text{0}9*\left(L_{\lambda },N_{x},N_{y},N_{z},P_{\lambda },S_{\lambda },M_{x},M_{y},M_{z},O_{\lambda },A_{\lambda },E_{\lambda },T_{\lambda },C_{\lambda },D,Q,V\right)\\ \text{0}1*\left({\left(r_{k},D_{2},R_{\left(\lambda ,2D\right)},S_{2}\right)}_{xoz},0.1*{\left(r_{k},D_{2},R_{\left(\lambda ,2D\right)},S_{2}\right)}_{yoz},0.1*{\left(r_{k},D_{2},R_{\left(\lambda ,2D\right)},S_{2}\right)}_{xoy}\right. \end{array}\right]. \end{array}$$

In the large-scale 3D point cloud classification architecture of MFOC-CliqueNet designed in this paper, the optimal combination matrix *Z*_0_ (MFOC) of multidimensional features of different label categories is visually displayed for observation, as shown in Figure 6.

### 4.6. Number of Training Epochs

An epoch refers to the process of sending all the data set sent to the network to complete a forward calculation and back propagation. As the number of epochs increases, the number of weight update iterations in the neural network will also increase. However, if there are too many epochs, it is prone to over-fitting. Conversely, too few training rounds will cause convergence to be too slow and not optimal state. Therefore, in order to make the MFOC-CliqueNet, in this paper achieve a good fitting state, the number of epochs is very important. Here, this paper makes an experimental comparison of different epoch numbers to get an efficient classification for large-scale 3D point cloud. The experimental results are shown in Table 6.

As can be seen from the above table, with the training epoch increases from 160, 200, and 250 to train the MFOC-CliqueNet network in this paper, the accuracy of each type of point cloud classification and the overall training accuracy are also improved accordingly.

### 4.7. Comparison of Results and Discussion

At present, many researchers at home and abroad have carried out large-scale point cloud classification research based on the Oakland point cloud dataset. Therefore, the method in this paper compares the classification accuracy with other methods based on this data set, as shown in Table 7. The experimental results show that the proposed method achieves an overall classification accuracy of 98.9% in Oakland point cloud dataset. Compared with our previous works [18], the overall classification accuracy is improved by 4.05%. And compared with papers [25–29], the overall classification accuracy has increased by 7.14%, 5.27%, 4.12%, 3.3%, 1.8%, and 1.21%, respectively.  Figure 7 shows the contrast effect of three-dimensional point cloud visualization in a large scene, Figure 7(a) is the visualization of the real-world data set, and Figure7(b) is the visualization of the classification results of the algorithm in this paper. In this paper, all point clouds in a large scene are projected in three directions: *XOY*, *YOZ*, and *XOZ*, and the overall classification accuracy is significantly better than other methods. For pole classification, *XOY* direction projection will affect the information feature extraction, resulting in poor classification efficiency of this category. At the same time, for wire classification, it is also affected by the *XOZ* direction projection, and making the classification efficiency not optimal. However, for the other three categories of objects, due to the projection in different directions, the self-occlusion and occluded of the 3D point cloud data itself are minimized, and more complete feature information of these point can be obtained, thereby improving the classification accuracy of these categories.

In the next work, we will improve the MFOC-CliqueNet further. Aiming at the situation that the geometric characteristics of some object categories in the 3D scene cloud data are close, such as pole and wire, we will improve the feature extraction efficiency of these two types of objects. Not only to improve the classification accuracy but also to enhance the robustness and generalization of MFOC-CliqueNet.

## 5. Conclusions

In the study of large-scene 3D point clouds, we introduce a new network structure MFOC-CliqueNet, based on the optimal combination of multidimensional features, which constructs the optimal combination matrix of multidimensional features by extracting the 3D features of 3D point cloud and the 2D features of multiple projection directions. CliqueNet is introduced into 3D point cloud data processing for the first time. It used a fixed number of parameters to obtain deeper representation space and combined with cyclic feedback to achieve the attention mechanism. It gets the MFOC with higher feature quality and passes it to the next Block by performing twice parameter cycle alternately update processing. At the same time, the multiscale feature strategy is adopted to effectively avoid the linear growth of parameters. The experiments show that we proposed MFOC-CliqueNet can reach the best level with fewer parameters, especially the total classification accuracy on the Oakland 3D large-scale point cloud data set reaches 98.9%. Different from the previous network, the proposed MFOC-CliqueNet provides the potential of the model development for other computer vision tasks in the future, especially for the application of increasing 3D data, such as semantic segmentation and salient objects detection of video, point cloud, remote sensing data [29].

## Figures and Tables

**Figure 1:** MFOC-CliqueNet: a large-scene 3D point cloud classification architecture based on optimal combination of multidimensional features. i = *B*, *C*, *D* in *Xi*, respectively, represent two-dimensional projection surfaces *XOY*, *YOZ*, *XOZ*; {*XD*, *XC*, *XB*} are the optimal arrangement and combination of two-dimensional features. The MFOC represents the optimal combination of multidimensional features.

**Figure 2:** Two-dimensional projection planes.

**Figure 3:** Visualization of point cloud projection in the three directions of *XOY*, *YOZ*, and *XOZ*: (a) left view; (b) rear view; (c) top view.

**Figure 4:** TBlock.

**Figure 5:** Comparison of different settings: (a) comparison of different initial learning rate. The initial learning rate of 1*e* − 3 is more conducive to the improvement of classification accuracy. (b) Comparison of different optimizer; optimizer moment is better than optimizer stochastic gradient descent (SGD) and adaptive moment estimation (adam).

**Figure 6:** MFOC of different label categories (input *Z*0 of the first clique block): (a) pole; (b) vegetation; (c) wire; (d) ground; (e) facade.

**Figure 7:** Visualization of classification results from ground truth and our MFOC-CliqueNet: (a) real-world labels of test data subsets and (b) point cloud classification results using our MFOC-CliqueNet.

**Table 1:** MFOC-CliqueNet network design.

Layer	*S*			
Convolution	Conv (5 × 5), 64, stride 2			
Pooling	Max pool (3 × 3), stride 2			
Block 1	36 × 5	36 × 5	36 × 5	40 × 6

Transition: conv (1 × 1), avg pool (2 × 2)				
Block 2	64 × 6	80 × 6	80 × 5	80 × 6

Transition: conv (1 × 1), avg pool (2 × 2)				
Block 3	100 × 6	120 × 6	150 × 6	160 × 6

Transition: conv (1 × 1), avg pool (2 × 2)				
Block 4	80 × 6	100 × 6	120 × 6	160 × 6

**Table 2:** Number of samples per class for the Oakland 3D point cloud data set.

Category	Training data	Test data
Vegetation	14441	257953
Wire	2571	3469
Pole	1086	7648
Ground	14121	930946
Facade	4713	109954
Sum	36932	1309970

**Table 3:** Classification results of different arrangements (%).

Order	Class					
	Pole	Vegetation	Wire	Ground	Facade	OA
DCB	0.127	0.723	**0.608**	0.946	**0.719**	**0.977**
CBD	0.012	0.821	0.351	0.883	0.190	0.973
CDB	0.088	**0.880**	0.555	**0.983**	0.418	0.975
DBC	**0.135**	0.796	0.422	0.980	0.426	0.959
BDC	0.022	0.833	0.206	0.765	0.340	0.958
BCD	0.043	0.843	0.305	0.938	0.167	0.947

The bold values indicate that the classification accuracy is the highest in the same category.

**Table 4:** Weighted combination results of multidimensional features (%).

3D : 2D	Class					
	Pole	Vegetation	Wire	Ground	Facade	OA
0.9 : 0.1	0.028	**0.965**	0.190	0.979	0.716	**0.9822**
0.8 : 0.2	0.032	0.902	0.299	0.962	0.475	0.9762
0.7 : 0.3	0.083	0.837	0.555	0.935	0.474	0.9744
0.6 : 0.4	0.039	0.812	0.407	0.971	0.594	0.9801
0.4 : 0.6	0.025	0.803	0.232	0.913	0.853	0.9724
0.3 : 0.7	0.135	0.677	0.299	0.982	0.842	0.9783
0.2 : 0.8	0.023	0.777	0.678	0.981	0.615	0.9750
0.1 : 0.9	0.076	0.519	0.276	0.977	0.907	0.9690

The bold values mean optimal overall classification results after weighted combination of multidimensional features of point cloud.

**Table 5:** Feature amplification results (%).

3D : 2D	Class					
	Pole	Vegetation	Wire	Ground	Facade	OA
1 : 2	0.047	0.717	0.403	0.985	0.628	0.9518
2 : 1	0.008	0.924	0.185	0.882	0.128	0.9664
1 : 1	0.127	0.723	0.608	0.946	0.719	0.9748
0.9 : 0.1	0.028	0.965	0.190	0.979	0.716	0.9822

**Table 6:** Feature amplification results (%).

Epoch	Class					
	Pole	Vegetation	Wire	Ground	Facade	OA
160	0.154	0.958	0.523	0.989	0.568	0.9798
200	0.028	0.965	0.190	0.979	0.716	0.9822
250	**0.160**	0.898	**0.591**	**0.995**	**0.946**	**0.9880**

**Table 7:** Methods comparison accuracy (%).

Class	Method					
	Pole	Vegetation	Wire	Ground	Facade	OA
M3N [23]	28.7	97.4	12.5	98.2	90.8	91.66
Literature [24]	22.3	90.7	5.3	99.6	87.6	93.53
Literature [25]	70.11	80.55	93.08	98.22	70.95	94.68
FDM [18]	68.42	80.68	92.93	98.37	71.13	94.75
CRFoptN [26]	59.7	92.0	10.7	99.9	94.6	95.5
MRF [27]	68.0	95.5	51.3	98.4	92.9	97.0
CCM [28]	82.67	97.83	30.26	99.17	90.33	97.59
Our method	16.0	89.8	59.1	99.5	**94.6**	**98.9**

Bold values highlight the advantages of our method and other literature methods in classification accuracy comparison.

## Data Availability

The data are included in the following link: http://www.cs.cmu.edu/∼vmr/datasets/oakland_3d/cvpr09/doc/
